The article "Effect and Significance of High-Quality Nursing on Blood Glucose, Pregnancy Outcome, and Neonatal Complications of Patients with Gestational Diabetes Mellitus" was retracted in 2023. Reasons: signs of a paper mill; compromised peer review; unreliable results or conclusions.

# Effect and Significance of High-Quality Nursing on Blood Glucose, Pregnancy Outcome, and Neonatal Complications of Patients with Gestational Diabetes Mellitus

**DOI:** 10.1155/2022/2426417

**Published:** 2022-04-26

**Authors:** Wenjuan Zhong, Chunxia Li, Jing Liu, Jinman Zhou, Zhong Xiao, Cuimei Li, Hui Wu

**Affiliations:** ^1^Pediatrics, Wuhan Wuchang Hospital, Wuchang Hospital Affiliated to Wuhan University of Science and Technology, Wuhan 430063, China; ^2^Department of Obstetrics and Gynecology, Wuhan Wuchang Hospital, Wuhan 430063, China; ^3^Nursing Department, Wuhan Wuchang Hospital, Wuhan 430063, China; ^4^General Surgery, Wuhan Wuchang Hospital, Wuhan 430063, China

## Abstract

**Objective:**

To explore the role of high-quality nursing on blood glucose, pregnancy outcome, and neonatal complications in patients with gestational diabetes mellitus.

**Methods:**

Altogether, 148 patients with GDM admitted to our hospital were selected as the research participants, 83 of whom received high-quality nursing as the observation group (OG). Another 65 patients received only routine care as the control group (CG). The blood sugar level, blood pressure value, and adverse pregnancy outcomes of the OG and the CG of patients after intervention were compared. The changes of psychological state and nursing satisfaction of the OG and the CG of patients were observed. The blood lipid level and neonatal complications of the OG and the CG were detected.

**Results:**

The blood sugar level of the OG was lower than that of the CG (*P* < 0.05). The systolic pressure and diastolic pressure of patients in the OG were lower than those in the CG after nursing intervention (*P* < 0.05). The abnormal delivery rate in the CG was evidently higher than that in the OG (*P* < 0.05). After intervention, SAS and SDS scores in the OG were lower than those in the CG (*P* < 0.05). The number of people who needed improvement and were dissatisfied in the OG was evidently lower than that in the CG (*P* < 0.05). TG and LDL-C in the OG were lower than those in the CG (*P* < 0.05). The total incidence of complications in the CG was evidently higher than that in the OG (*P* < 0.05).

**Conclusion:**

High-quality nursing can reduce blood sugar and blood pressure of GDM patients and has a great protective effect on maternal and infant health, which is worthy of clinical practice.

## 1. Introduction

Gestational diabetes mellitus (GDM) is the first diabetes mellitus due to abnormal maternal glucose metabolism after pregnancy, which is one of the common complications during pregnancy [1]. Pregnant women with GDM often have no obvious symptoms, and sometimes, fasting blood glucose may be normal, which may easily lead to missed diagnosis and delay the treatment of pregnant women [2]. GDM is easy to cause maternal infection, polyhydramnios, and hypertension [3], and it is easy to cause a series of complications such as fetal hyperglycemia, hyperinsulinemia, macrosomia, and neonatal hypoglycemia [4]. In recent years, with the rapid development of society, the living standard of the people is continuously improving, the number of elderly women in gynecology is increasing, the number of GDM patients is increasing evidently [5], and the incidence of complications related to newborn babies is also increasing gradually, which seriously threatens the life safety of mothers and infants [6]. At present, the doctors for GDM will first suggest patients to undergo diet therapy and exercise therapy [7] to maintain the blood sugar of GDM patients in the normal range. If the blood sugar is still poorly controlled, insulin will be used for treatment [8]. However, drug use may cause adverse effects on the fetus [9]. Therefore, it is particularly important to take effective intervention measures for mothers and children in advance and to carry out scientific diet guidance and other aspects of intervention, so as to reduce complications of mothers and children and reduce neonatal mortality.

The article "Effect and Significance of High-Quality Nursing on Blood Glucose, Pregnancy Outcome, and Neonatal Complications of Patients with Gestational Diabetes Mellitus" was retracted in 2023. Reasons: signs of a paper mill; compromised peer review; unreliable results or conclusions.

Previous studies have pointed out that the intervention of nursing methods can effectively improve the complications of GDM patients. For example, Tang [10] showed that detailed consultation and guidance by professional medical personnel are useful for improving the condition of GDM patients. It can be seen that nursing methods have a key positive effect on GDM patients and infants [11]. The “high-quality nursing service demonstration project” is an important guiding measure for the reform of nursing work in our country at present [12] and is also an important measure for establishing a patient-centered nursing service concept in China [13]. Previous studies have suggested that high-quality nursing can effectively reduce the blood sugar of patients by guiding their diet and exercise [14]. However, less attention has been paid to the complications of the delivered babies. Therefore, in order to ensure the positive effect of high-quality nursing on GDM patients and newborns, this study explored the role of high-quality nursing on the blood glucose level, pregnancy outcome, and neonatal complications of GDM patients, providing effective reference and guidance for future clinical nursing intervention on GDM.

## 2. Data and Methods

### 2.1. General Data

Altogether, 148 GDM patients from July 2017 to July 2019 were obtained as research participants, 83 of whom received high-quality nursing as the observation group (OG). Another 65 patients received routine nursing as the control group (CG). This experiment has been approved by the Ethics Committee. All the patients have signed informed consent forms.

The article "Effect and Significance of High-Quality Nursing on Blood Glucose, Pregnancy Outcome, and Neonatal Complications of Patients with Gestational Diabetes Mellitus" was retracted in 2023. Reasons: signs of a paper mill; compromised peer review; unreliable results or conclusions.

### 2.2. Inclusion and Exclusion Criteria

*Inclusion criteria*: all participants were diagnosed as GDM in our hospital and were pregnant for the first time; after diagnosis, all patients were treated in our hospital and had complete clinical data; all patients agreed to cooperate with the medical staff and signed the informed consent form.

*Exclusion criteria*: patients with other malignant tumors, patients with multiple chronic diseases, patients with other cardiovascular and cerebrovascular diseases, patients with organ dysfunction, patients with drug allergies, patients with mental diseases or physical disabilities who could not take care of themselves, and referred patients were excluded.

### 2.3. Treatment Methods

The CG adopted the routine nursing mode, and the head nurse deployed the nursing staff and carried out the oral doctor's advice process, including providing health guidance to the patients, closely observing the changes in blood sugar, and requiring the patients to undergo regular prenatal examination every month. The OG implemented high-quality nursing based on the CG. First, the nurses should comprehensively understand the condition of the patients and examined them. According to the blood sugar level of the patients, different diet plans were designated, health education was actively carried out for the patients and their families, diet intervention was applied for the patients, and blood sugar was controlled. The nursing staff should ensure the nutritional needs of pregnant women and supplement trace elements and vitamins. A reasonable exercise plan was conducted for patients to actively encourage patients to take appropriate exercise, thus reducing the patient's body mass and improving insulin sensitivity as far as possible with safety. At the same time, psychological counseling should be carried out for patients to understand the causes of related diseases and inform the treatment methods so as to improve the treatment compliance of patients and eliminate their negative psychology such as tension, anxiety, and fear. Regular health examination was performed for patients.

### 2.4. Outcome Measures

The blood sugar level, blood pressure value, and adverse pregnancy outcomes of the OG and the CG of patients after the intervention were compared. The psychological state and satisfaction of the OG and the CG were observed. Total cholesterol (TC), triglyceride (TG), low-density lipoprotein cholesterol (LDL-C), high-density lipoprotein cholesterol (HDL-C), and neonatal complications were detected.

The article "Effect and Significance of High-Quality Nursing on Blood Glucose, Pregnancy Outcome, and Neonatal Complications of Patients with Gestational Diabetes Mellitus" was retracted in 2023. Reasons: signs of a paper mill; compromised peer review; unreliable results or conclusions.

### 2.5. Statistical Method

SPSS22.0 was applied to make statistical analysis on the data results and GraphPad7 to visualize graphs on the data results. The counting data were represented by rate, and the chi-squared test was applied for comparison. The measurement data were represented as the mean ± standard deviation, and the comparison adopted the *t*-test. *P* < 0.05 means the difference was statistically evident.

## 3. Results

### 3.1. Blood Sugar Level of Two Groups of Patients after Nursing Intervention

The blood glucose levels of the OG and the CG of patients after intervention were compared. The results showed that the fasting blood glucose of the patients in the OG was lower than that of the patients in the CG two hours after breakfast, two hours after lunch, and two hours after dinner (*P* < 0.05). All the data are indicated in Figure 1.

### 3.2. Comparison of Blood Pressure of the OG and the CG after Intervention

The blood pressure values of the OG and the CG of patients after the intervention were compared. The results showed that the systolic pressure and diastolic pressure of the patients in the OG were lower than those in the CG after nursing intervention (*P* < 0.05). All the data are indicated in Figure 2.

### 3.3. Adverse Pregnancy Outcomes of Two Groups of Patients

The adverse pregnancy outcomes of the OG and the CG were recorded. The results showed 76 cases of normal delivery in the OG and 65 cases of normal delivery in the CG, the total abnormal delivery rate in the OG was 8.43%, the total abnormal delivery rate in the CG was 24.62%, and that in the CG was evidently higher than that in the OG (*P* < 0.05). All the data are indicated in Table 1.

### 3.4. Changes of Psychological State in Two Groups of Patients

There was no evident difference in SAS and SDS scores between the OG and the CG before intervention (*P* > 0.05). The SAS scores in the OG after intervention were evidently lower than those in the CG after intervention (*P* < 0.05). The SDS score of OG after intervention was also evidently lower than that of CG after intervention (*P* < 0.05). After intervention, SAS and SDS scores of the OG and the CG were evidently lower than that before intervention (*P* < 0.05). All the data are indicated in Figure 3.

### 3.5. Comparison of Nursing Satisfaction between the OG and the CG

Comparing nursing satisfaction, we found that the total satisfaction of patients in the OG was 95.18 and that in the CG was 66.15. The number of patients who needed improvement and were not satisfied in the OG was evidently lower than that in the CG (*P* < 0.05). All the data are indicated in Table 2.

The article "Effect and Significance of High-Quality Nursing on Blood Glucose, Pregnancy Outcome, and Neonatal Complications of Patients with Gestational Diabetes Mellitus" was retracted in 2023. Reasons: signs of a paper mill; compromised peer review; unreliable results or conclusions.

### 3.6. Blood Lipid Level of Newborns in Two Groups

The blood lipid levels of newborns in the two groups were detected. The results showed that the TG and LDL-C levels of newborns in the OG were evidently lower than those in the CG (*P* < 0.05), while the TC and HDL-C levels of newborns in the two groups had no evident difference (*P* > 0.05). All the data are indicated in Figure 4.

### 3.7. Incidence of Neonatal Complications in Two Groups

The results showed that the total incidence rate of neonatal complications in the OG was 16.87%, that in the CG was 35.38%, and that in the CG was evidently higher than that in the OG (*P* < 0.05). All the data are indicated in Table 3.

## 4. Discussion

GDM seriously affects the health of the mother and infant [15]. Studies have confirmed that GDM is an independent risk factor for adverse pregnancy outcomes [15]. And some patients with GDM will be affecting their life, thus reducing the quality of life of patients [16]. At present, the pathogenesis of GDM is not completely clear. The self-blood sugar control effect of patients is not ideal; the weight increases rapidly, thus increasing the risk of adverse pregnancy outcomes; and patients are often accompanied by different degrees of negative psychology, which is harmful to fetal health [17]. How to effectively control the blood sugar level of pregnant and lying-in women has always been the research focus of obstetrics doctors. Modern medical research showed that the blood sugar level of GDM patients was closely related to their life and eating habits [18]. However, nursing intervention is applied with the concept of patient-centeredness, and high-quality nursing intervention is very important for patients' recovery and health [19]. Therefore, this study explored the influence of high-quality nursing intervention on the blood glucose level, pregnancy outcome, and neonatal complications of gestational diabetes mellitus patients.

Our current results showed that the fasting blood glucose of the patients in the OG was lower than that of the CG two hours after breakfast, two hours after lunch, and two hours after dinner, and the systolic blood pressure and diastolic blood pressure of the patients in the OG are lower than that of the CG after nursing intervention. We investigated the adverse pregnancy outcomes of the OG and the CG. The results revealed that there were 76 normal deliveries in the OG, 65 normal deliveries in the CG, 4 polyhydramnios, 2 oligohydramnios, 1 premature rupture of membranes in the OG, 8 polyhydramnios, 3 oligohydramnios, 2 premature rupture of membranes, and 3 postpartum hemorrhage in the OG. The abnormal delivery rate in the CG was evidently higher than that in the OG. This suggested that the implementation of high-quality care is of great significance for lowering blood sugar and improving blood pressure of patients. The application of high-quality nursing intervention can reduce adverse pregnancy outcomes of GDM patients and greatly reduce delivery complications of patients [20]. This is also consistent with the effect of high-quality nursing intervention mentioned by previous studies. For example, the research of Beets et al. [21] showed that high-quality nursing intervention is of great significance to the recovery of colorectal cancer patients. However, Metzger et al. [22] confirmed that high-quality nursing intervention had an important impact on adverse pregnancy outcomes of GDM patients. Then, we investigated the SDS and SAS scores and nursing satisfaction of the OG and the CG. The results showed that the SDS and SAS scores of the OG were evidently lower than those of the CG, and the nursing satisfaction of the OG was higher than that of the CG. It further indicated that high-quality nursing intervention can reduce negative emotions and improve satisfaction. Furthermore, studies have also proved that high-quality nursing has better clinical application value, so it is not repeated here. All the above studies have confirmed the important clinical application significance of nursing intervention in the operation. However, we speculated that its value is mainly reflected in the following aspects: (1) The level of adrenocortical hormone, anterior pituitary hormone, and other antagonistic insulin hormones in pregnant women during pregnancy increased. Endocrine changes affected the glucose metabolic pathway, leading to an increase in blood sugar. Hyperglycemia in the body would destroy the body system, leading to pathological changes and various complications [23]. The blood sugar level of patients was closely related to diet, and the change of diet was closely related to blood sugar [24]. However, high-quality nursing staff would formulate a special diet plan according to the different conditions of pregnant women, so as to make the diet more reasonable and balanced, adjust the diet structure, and thus reduce the blood sugar of patients. (2) GDM was closely related to hypertension. The occurrence of GDM would greatly induce the risk of complications such as hypertension and lead to a variety of adverse pregnancy outcomes [7]. High-quality nursing was based on the scientific nursing mode, which continuously carried out standardized nursing operations for patients. The blood sugar of patients decreased, and the blood pressure immediately decreased. Through nursing methods, patients have mastered certain disease knowledge and improved treatment compliance, thus reducing adverse pregnancy outcomes of patients. (3) Complications of GDM, obesity, and diet problems were easy to create negative emotions for patients, while negative emotions could directly aggravate the illness, and even postpartum depression in severe cases [25]. High-quality nursing intervention would eliminate the anxiety and fear of patients through continuous communication with patients, which is of great help to the health of the mother and fetus. In addition, the comfort of the parturient was increased, the blood sugar was reduced, the incidence rate of adverse reactions of the parturient was reduced, and the nursing satisfaction degree was also improved. In order to further clarify the positive significance of high-quality nursing for GDM, we have made statistics on complications of infants delivered by GDM parturients. The results show that the total incidence rate of neonatal complications in the OG was evidently lower than that in the CG. The results showed that the TG and LDL-C levels of newborns in the OG were evidently lower than those in the CG, and there was no evident difference in TC and HDL-C levels. Whether the fetus can obtain nutrition smoothly in the maternal blood mainly depends on the changes of blood lipid metabolism, while abnormal changes in blood pressure and blood glucose will affect the changes of fetal blood lipid, resulting in an increased risk of damage to maternal and infant health [26]. This result further supported the above experiment, which showed that high-quality nursing had a very important influence on GDM parturient and fetus.

The article "Effect and Significance of High-Quality Nursing on Blood Glucose, Pregnancy Outcome, and Neonatal Complications of Patients with Gestational Diabetes Mellitus" was retracted in 2023. Reasons: signs of a paper mill; compromised peer review; unreliable results or conclusions.

The purpose of our current study was to explore the application value of high-quality nursing intervention to GDM, but there are still deficiencies due to limited experimental conditions. For example, there are many nursing methods in clinical practice, but there is still great controversy over the choice of the best nursing mode for GDM. In addition, only routine nursing is used as a control in this article, and it is not excluded that the application of high-quality nursing intervention may differ from the results of this study when compared with other nursing modes. Moreover, the current study is short in duration, and the long-term prognosis is not clear yet, which still requires further analysis. Furthermore, we will expand the sample size of our study, extend the study period, and conduct more detailed and comprehensive experimental analysis to obtain more perfect results.

To sum up, high-quality nursing can reduce blood sugar and blood pressure of GDM patients and has a great protective effect on maternal and infant health, which is worthy of clinical use.

The article "Effect and Significance of High-Quality Nursing on Blood Glucose, Pregnancy Outcome, and Neonatal Complications of Patients with Gestational Diabetes Mellitus" was retracted in 2023. Reasons: signs of a paper mill; compromised peer review; unreliable results or conclusions.

## Figures and Tables

**Figure 1:** Blood sugar level of two groups of patients after nursing intervention. Note: ∗ indicates *P* < 0.05.

**Figure 2:** Blood pressure values of two groups of patients after nursing intervention: (a) systolic blood pressure comparison between the OG and the CG after nursing intervention; (b) comparison of diastolic blood pressure between the OG and the CG after nursing intervention. Note: ∗ indicates *P* < 0.05.

**Figure 3:** Changes in the psychological state of two groups of patients: (a) SAS scores before and after intervention in both groups: (b) SDS score before and after intervention in both groups. Note: ∗ indicates *P* < 0.05.

**Figure 4:** Comparison of blood lipid level between two groups of newborns: (a) comparison of TC between two groups of patients; (b) comparison of TG between the OG and the CG; (c) comparison of LDL-C levels between the OG and the CG; (d) comparison of HDL-C levels between the OG and the CG. Note: ∗ indicates *P* < 0.05.

**Table 1:** Adverse pregnancy outcomes.

	OG (*n* = 83)	CG (*n* = 65)	*χ* ^2^	*P*
Normal delivery	76 (91.57)	49 (75.38)		
Abnormal delivery				
Polyhydramnios	4 (4.82)	8 (11.76)		
Oligohydramnios	2 (2.41)	3 (4.62)		
Premature rupture of membranes	1 (1.20)	2 (3.08)		
Postpartum hemorrhage	0 (0.00)	3 (4.62)		
Total rate (%)	7 (8.43)	16 (24.62)	7.272	0.007

**Table 2:** Comparison of nursing satisfaction between two groups of patients.

	OG (*n* = 83)	CG (*n* = 65)	*χ* ^2^	*P*
Very satisfied	60 (72.29)	18 (27.69)		
Satisfied	19 (22.89)	25 (38.46)		
Need improvement	3 (3.61)	15 (23.08)		
Dissatisfied	1 (1.20)	7 (10.77)		
Total satisfaction (%)	79 (95.18)	43 (66.15)	21.210	<0.001

**Table 3:** Incidence of neonatal complications in two groups.

	OG (*n* = 83)	CG (*n* = 65)	*χ* ^2^	*P*
Infection	2 (2.41)	5 (7.69)		
Hypoglycemia	4 (4.82)	6 (9.23)		
Asphyxia	2 (2.41)	3 (4.62)		
Macrosomia	4 (4.82)	5 (7.69)		
Hyperbilirubinemia	1 (1.20)	2 (3.08)		
Respiratory distress syndrome	1 (1.20)	2 (3.08)		
Total incidence (%)	14 (16.87)	23 (35.38)	6.666	0.010

## Data Availability

Our data are real and available, and you can find them in our hospital database.
